# Analysis of College Students' Network Moral Behavior by the History of Ideological and Political Education under Deep Learning

This article has been retracted.

**DOI:** 10.1155/2022/9885274

**Published:** 2022-08-12

**Authors:** Yin Zhang

**Affiliations:** Department of History, Hebei University, Baoding 071000, Hebei, China

## Abstract

The research on the history of ideological and political education (IPE) is the basis for deepening it, and it is also of great help to higher education. The diversity of network information also easily leads to poor guidance for college students who are not strong in discrimination. This study adopts the method of a questionnaire survey to investigate the common moral anomie among college students in the network space. The survey data are sorted and classified and then input into the recurrent neural network structure for data analysis using deep learning (DL) algorithms. The results are fed back to the investigators intuitively and understandably. The results show that some college students have some problems, such as lack of network moral knowledge, vague values, moral behavior anomia, spatial knowledge and behavior inconsistency, and moral and emotional indifference. DL algorithms are added to the analysis process to make the findings more objective. These conclusions provide reference suggestions for subsequent research on college students' online moral behavior in the context of IPE history.

## 1. Introduction

The history of ideological and political education (IPE) has a special status in its discipline and plays an irreplaceable basic role [1]. IPE is an important part of Chinese college education, which plays an important role and significance in improving the ideological and political level and moral cultivation of contemporary college students [2]. General Secretary Xi Jinping emphasized that IPE should run through the whole process of education and teaching. It should not only run through the education from beginning to end but also implement the students' growth and talent from beginning to end. Although the quality of IPE work in colleges and universities has improved, there are still weak links that need to be improved [3]. Especially with the development of the Internet, whether the online moral behavior of college students is standardized has also attracted the attention of the state. On February 3, 2015, China Internet Network Information Center released the 35th Statistical Report on Internet development in China. The report shows that as of December 2014, Chinese netizens reached 649 million. Students are still the largest group of Chinese netizens, accounting for 23.8%. From the research report on Internet behavior of Chinese youth in 2014, the weekly online time of college netizens increased to 25.9 hours, an increase of 0.9 hours over the previous year. College students are the largest and most active group of Chinese netizens [4]. College students' world, life, and values outlook are not fully mature, and they are easily affected by some bad factors and have network moral problems. Therefore, research on college students' network moral security behavior is necessary [5].

Usually, in order to understand and deeply analyze the thoughts or mental health of college students, scholars use questionnaires to collect relevant data. They combine some data processing techniques to dig out the underlying patterns in the data. Educators can formulate some strategies for assistance and improvement based on the final analysis results. Ilieva et al. evaluated the impact of COVID-19 on college students' learning and collected information and data on college students' attitudes toward distance learning by issuing questionnaires. They proposed a new frame of reference for educational data processing. The framework combines machine learning, multicriteria decision-making, and big data techniques with information symmetry and asymmetry [6]. Taeymans et al. distributed a questionnaire to university students to explore whether college students' lifestyle of studying during the outbreak of COVID-19 is healthy. They analyzed the questionnaire data using frequency analysis and nonparametric statistical methods [7]. Fook et al. pointed out that since smartphone users include students from middle school to university, frequent use of mobile phones will lead to mobile phone dependence. This phenomenon can negatively impact the academic performance. Therefore, college students' smartphone use, time spent, factors, and activities involved were investigated, and the possible risks of college students' mobile phone addiction were demonstrated. Data analysis was performed using descriptive statistical methods such as mean, standard deviation, frequency, and percentage [8]. Shen et al. studied gender differences in the prevalence, risk factors, and clinical correlates of Internet addiction among Chinese college students. The method of cross-sectional design and convenience sampling was adopted to investigate 8,098 college students in the human province [9].

In the past two years, scholars' exploration of college students' behavior has mainly focused on the physical and mental health status under the influence of COVID-19 and the investigation of the reasons for using electronic products or Internet addiction. Data processing uses some relatively simple statistical methods. However, with the rapid development of information technology, there are more and more ways for college students to obtain information. Students are also increasingly affected by bad information on the Internet. These electronic products will make students prone to some problems of online moral behavior anomie. Therefore, some more effective technical means have been adopted to conduct in-depth research on college students' online moral behavior. The innovative point is starting from the historical development of IPE, using the questionnaire survey and CNN with good time-series data processing ability. The current situation of college students' online moral behavior is analyzed, and the survey results are presented objectively and clearly through CNN. The algorithm makes the research results more accurate and increases the credibility. Based on the development history of IPE, the analysis of college students' online moral behavior has certain feasibility. There are few achievements in introducing algorithms in this research direction, which can provide a reference for subsequent research in similar directions.

## 2. Methods

### 2.1. Analysis of Deep Learning Algorithms

Geoffrey Hinton first proposed deep learning (DL) in the journal Science, and it was studied by later generations and gradually emerged. DL research extends the original basis of machine learning [10]. Compared with the machine learning network, the DL network optimizes the hierarchical data of the network structure, making the overall structure more complex. The internal operation algorithm has also undergone greater progress [11, 12].

DL learns the inherent laws and representation levels of sample data by analyzing the underlying laws and data structure levels within the sample data. The data obtained during the learning process are used to provide reference interpretations to data in other domains [13]. Initially, the research goal of DL algorithms was to be used in the field of artificial intelligence (AI), helping AI to have the ability to analyze and learn like humans and to recognize various forms of data. DL has achieved results in many fields. The analysis and learning ability of AI is improved through DL, thereby helping humans solve many complex data research problems [14].

DL is a general term for data research models and methods, and DL is classified according to specific research content. The classification results are shown in Table 1 [15].

#### 2.1.1. CNN

CNN is a kind of artificial neural network, which is often used in speech analysis and image recognition, and the recognition and the analysis effect is accurate and direct, so it has been widely used [16]. The internal structure of CNN is like the biological neural network. A new weight-sharing network structure is constructed by reducing the complexity of the network structure and reducing the input weights of the model input layer. The difference between CNN and ordinary neural networks is that CNN contains a feature extractor composed of convolutional and subsampling layers. In a convolutional layer of a CNN, a neuron is only connected to some of its neighbours. A convolutional layer of CNN usually contains several feature maps. Each feature plane consists of some neurons arranged in a rectangle, and neurons in the same feature plane share weights. Here, the shared weights are the convolution kernels. The convolution kernel is usually initialized in the form of a random decimal matrix. During the training process of the network, the convolution kernel will learn to obtain reasonable weights. The immediate benefit of sharing weights (convolution kernels) is to reduce the connections between the layers of the network, which in turn reduces the risk of overfitting.

Subsampling is also called pooling, and there are usually two forms of mean subsampling and max pooling. Subsampling can be seen as a special kind of a convolution process. Convolution and subsampling greatly simplify model complexity and reduce model parameters. When the input image is a multidimensional layer, it is directly input into the algorithm structure, which saves the complicated analysis time and improves the algorithm's efficiency [17]. Additionally, CNN also has the advantage of high efficiency in training weights. For example, in the traditional neural network structure, the neuron structure of the upper and lower layers is connected to form a whole. In the process of training the weights, the parameter values that need to be trained are doubled. As for the CNN structure, it shares image data input inside the structure to each neuron through the internal “convolution kernel” as the intermediary between upper and lower neurons and maintains the original location structure after neural network processing. Therefore, a CNN is more akin to a special multilayer perceptual device that recognizes the structure of a two-dimensional image. The network structure also enables CNN to effectively deal with many forms of image deformations [18].

CNN is a multilayer neural network. Its structure is shown in Figure 1.

In Figure 1, the basic operating units of CNN include convolution, pooling, full connection, and recognition operations. The operation principle and process of each unit are analyzed in detail.

Convolution operation: it uses the feature map of the previous layer to perform a convolution operation with a learnable convolution kernel. The output of the convolution result after the activation function forms this layer's neurons, thus forming the feature map of this layer, also known as the feature extraction layer. The input of each neuron is connected to the local receptive field of the previous layer, and the local features are extracted. Once the local feature is extracted, its positional relationship with other features is determined. The input image matrix and the subsequent convolution kernel and feature map matrix are square matrices. Suppose the input matrix size is *w*, the convolution kernel size is *k*, the stride is *s*, and the number of zero-padded layers is *p*. The feature size calculation after convolution is shown in the following equation (1) [19]:

(1) $$\begin{array}{c} w=\frac{\left(w+2p-k\right)}{s}+1. \end{array}$$

Pooling operation: it can aggregate features well and reduce dimensionality to reduce the amount of computation. The pooling operation divides the input signal into nonoverlapping regions, and the spatial resolution of the network is reduced by a pooling (downsampling) operation for each region. For example, max pooling is to select the maximum value in the area, and mean pooling is to calculate the average value in the area. This operation is used to remove skew and distortion from the signal [20].

Full connection operation: after the input signal undergoes multiple convolution kernel pooling operations, the extracted data features are mapped to the output layer to realize feature output. The output is multiple groups of signals. After the full connection operation, the multiple groups of signals are sequentially combined into a group of signals.

The operation of the input value of each convolutional layer is shown in the following equation:

(2) $$\begin{array}{c} V=conv2\;\left(W,\;X,\;valid\right)+b. \end{array}$$

In (2), *conv*2 is the function of convolution operation; the third parameter valid refers to the type of convolution operation; *b* is the bias [21]; *W* is the weight matrix; the weight matrix of each layer is different; and *X* is in matrix form.

The output is shown in the following equation:

(3) $$\begin{array}{c} Y=\varphi \left(V\right) \end{array}$$

In (3), *Y* is in matrix form. Assuming that the last layer of the connection layer is *L*, the total error is shown in the following equation:

(4) $$\begin{array}{c} E=\frac{1}{2}d-y_{L2}^{2}. \end{array}$$

where *d* is the variable that is expected to be output and *y* is the variable output by the CNN.

#### 2.1.2. DBN Analysis

DBN can be interpreted as a Bayesian probabilistic generative model consisting of multiple layers of random latent variables. The upper two layers have undirected symmetric connections, and the lower layers get top-down directed connections from the upper layer. The state of the bottommost unit is the visible input data vector. If DBN consists of a stack of 2F structural units, the structural unit is usually a restricted Boltzmann machine (RBM). In the stack, the number of visible layer neurons of each RBM unit is equal to the number of hidden layer neurons of the previous RBM unit. According to the DL mechanism, the input samples are used to train the first-layer RBM unit, and its output is used to train the second-layer RBM model. The RBM model is stacked to improve the model performance by adding layers. In the unsupervised pretraining process, after the DBN code is input to top-level RBM, the top-level state is decoded to the bottom-level unit to realize the reconstruction of the input. As the structural unit of DBN, RBM shares parameters with each layer of DBN [22]. DBN solves the optimization problem of deep neural networks by adopting layer-by-layer training. The layer-by-layer training gives the whole network better initial weights to reach the optimal solution only after fine-tuning. The essence of RBM is a powerful tool for supervised learning. It can be used to reduce the dimensionality of images with less hidden layer settings, learn to extract features for hidden layer output, auto encoder, and DBN stacked with multiple RBM, and so on.

#### 2.1.3. RNN

RNN is a special neural network structure mainly used to study temporal sequence-related problems. It has a tree-like hierarchical structure and can perform recursive operations on the input information of network nodes in the order of their connection. RNN is a composite neural structure composed of multiple layers of neural structures, and each layer has the same neural structure. Its input is two child nodes (or more than one), and the output is the parent node generated by encoding these two child nodes. The dimension of the parent node and each child node is the same data. After the input, the hidden neuron structure is repeated internally. The input is not only the real-time data but also the forgetting state of the previous stage [23]. RNN can encode a tree or graph structure information as a vector, mapping the information into a semantic vector space. This semantic vector space satisfies certain properties, such as semantically similar vectors being closer. The research of RNN started in the 1980s and developed into one of the DL algorithms in the early 2000s. Among them, bidirectional RNN (Bi-RNN) and long short-term memory (LSTM) networks are common RNN. The structure of RNN is shown in Figure 2 [24].

In Figure 2, the RNN will have an input *x*_*t*_ at every moment. Then, calculate the new state *h*_*t*_ according to the state *h*_*t*−1_ at the previous moment and output *O*_*t*_. The current state *h*_*t*_ of the RNN is jointly determined according to the state *h*_*t*−1_ at the previous moment and the current input *x*_*t*_. At the time *t*, the state *h*_*t*−1_ condenses the information of the previous sequence and is used as a reference for the output. Since the length of the sequence can be extended indefinitely, the *h* state with a limited dimension cannot save all the information of the sequence. Therefore, the model must learn to retain only the most important information related to the later tasks [25]. For any sequence time *t*, the hidden state *h*_*t*_ is calculated by *x*_*t*_ and *h*_*t*−1_, as shown in the following equation:

(5) $$\begin{array}{c} h_{t}=f\left(s^{t-1},\;x_{t},\theta \right). \end{array}$$

In equation (5), *s* is the internal state, *f* is the excitation function, and *θ* is the weight coefficient inside the cyclic unit. The calculation of the output value *O*_*t*_ at time *t* is shown in the following equation:

(6) $$\begin{array}{c} O_{t}=Vh_{t}+c. \end{array}$$

In equation (6), *V* and *c* are weight coefficients.

There are two ways to connect RNN: recurrent unit-recurrent unit connection and output node-recurrent unit connection.

(1) Cyclic unit-cycle unit connection is also known as “hidden-hidden connection (HHC)” or full connection. The state of the current time step of each recurrent unit is determined by the input and the state of the previous time node, as shown in the following equation:
  (7) $$\begin{array}{c} h_{t}=f\left(Uh_{t-1}+Wx_{t}+b\right). \end{array}$$
In (7), *U* and *W* are the weights of the loop nodes, the former is called the state-state weight, and the latter is called the state-input weight. A bidirectional RNN (BRNN) can be obtained by stacking forward and reversing recurrent unit-recurrent unit connections.
(2) Output node-cyclic unit connection: in this connection, the state of the recurrent unit is determined by the input of the time node and the output value of the previous time node [26], as shown in the following equation:
  (8) $$\begin{array}{c} h_{t}=f\left(Uo_{t-1}+Wx_{t}+b|.\right) \end{array}$$

### 2.2. Back Propagation through Time

Back propagation through time (BPTT) is an extension of the backpropagation algorithm combined with the RNN structure. The cyclic structure is decomposed into a layer structure by expanding the RNN structure. Each layer structure is calculated according to the framework of RNN. According to the parameter sharing nature of RNN, the gradient of the weight is the sum of all layers [27]. The loss function *L* operates as shown in the following equation:

(9) $$\begin{array}{c} L=-\sum_{t=1}^{\tau }logp\left(y^{\left(t\right)}|x_{1},\ldots ,x_{t}\right). \end{array}$$

The error *E* is shown in the following equation:

(10) $$\begin{array}{c} E=\frac{1}{2}\sum_{k=1}^{l}{\left[d_{k}-f\left(net_{k}\right)\right]}^{2}. \end{array}$$

RNN works with serialized structured data by connecting neurons into strings of structures. Each neuron can use internal variables to hold input sequence data previously. Therefore, the whole sequence is compressed into an abstract representation. The lower part of the data can be classified, or a new sequence can be generated according to this representation. Therefore, the RNN structure is often used to study time-related problems [28].

### 2.3. RNN's Analysis of College Students' Network Moral Behavior

Data acquisition: this study used a questionnaire survey method to collect data. Undergraduate students in the Baoding city are surveyed on the online moral behavior of college students, supplemented by discussions, oral surveys, and online surveys. In order to make the survey results more representative, the survey subjects cover a wide range of subjects, and the subjects of the questionnaires cover liberal arts, science, engineering, medicine, art, and other disciplines. A total of 220 questionnaires are distributed in this survey. Two hundred five questionnaires are recovered, there are 200 valid questionnaires, and the effective recovery rate is 90.9%. The details of the grade distribution of the survey respondents are shown in Figure 3.

In Figure 3, in this valid questionnaire, there are 43 freshmen, 43 sophomores, 52 juniors, and 62 seniors. The distribution of the surveyed subjects is uniform. The subjects of the survey are shown in Figure 4.

In Figure 4, among the respondents of this valid questionnaire, there are 50 people in the liberal arts department, 42 people in the science department, 38 people in the medical department, 36 people in the art department, and 34 people in the engineering department. The distribution of subjects is relatively even.

A questionnaire on the Internet morality of college students is compiled, which went through the preliminary drafting of questions, multiple revisions, small-scale testing, reexamination, and final drafting to ensure the credibility and validity of the survey results. There are 33 questions in the questionnaire, and the content mainly includes four aspects: (1) the basic information of the respondents, such as gender, grade, age, school type, and discipline; (2) the specific characteristics of the respondents, such as Internet access time, location, the purpose of surfing the Internet, network media, and network behavior; (3) respondents' views on certain online ethical issues, such as online speech, online pornography, network security, and network hacking; (4) respondents' views on certain online moral issues; the knowledge of online moral education, such as the way to carry out online moral education, and the methods and suggestions for improving the level of online moral education. Finally, the questionnaires are collected, checked, and organized by the research group members and then input into RNN for data analysis. The specific research process is shown in Figure 5.

In Figure 5, the research data are obtained through a questionnaire survey, and the data are organized and classified. Missing key data are completed and denoised. The processed data are input into RNN for operation, and the output results are sent to the user in a straightforward and easy-to-understand manner.

## 3. Results

### 3.1. Analysis of the Survey Results of Network Moral Education

At present, the survey of college students' views on online moral education is shown in Figure 6.

In Figure 6, 77.0% of the respondents believe that college students must receive online moral education. However, only 14.8% of the students said that they are very interested in the online moral education carried out by the school. As high as 80.1% of the respondents said, they did not care about the online moral education courses carried out by schools. Even 5.1% of the students said that they hated online education courses. As a result of this polarization, the cybersecurity education courses carried out by colleges and universities will have a little effect, and the contradictory attitude towards cybersecurity education will also lead to the lack of cybersecurity education knowledge.

The situation of the respondents receiving the education on online moral behavior is investigated, as shown in Figure 7.

In Figure 7, 18% of the respondents have received education on network ethics and security, 22.3% have only had access to the education on network security ethics, and 15.7% of the respondents have learned about relevant network security education norms. At present, the progress of China's cyber security ethics education is still relatively slow, and the proportion of educated people is relatively small. Governments and schools should step up efforts to popularize cybersecurity ethics.

### 3.2. Analysis of the Survey Results of Network Moral Values

The online moral values of college students are investigated, as shown in Figure 8.

In Figure 8, 55.2% of the respondents believe that browsing pornographic websites is not a wrong behavior. 24.6% believe that cyber hacking does not violate the law. 20.4% believe that the Internet human flesh search is reasonable and can help control bad behaviors and crimes. 39.2% believe that infringing on others' intellectual property rights on the Internet would not cause great losses. 35.8% believe that verbal attacks against others on the Internet did not matter because they did not know each other. 68.3% believe that online dating is also a way to find true love while also pursuing excitement and bringing new experiences. Most college students have incorrect views on online moral behavior, and the concept of online moral behavior is vaguely defined.

### 3.3. Analysis of the Survey Results of Network Moral Behavior

The online moral behavior of college students is investigated. The results are shown in Figure 9, contrasted with their perceptions of ethical behavior online.

In Figure 9, 42.5% of the respondents admitted that their behavior on the Internet is slightly inconsistent with their actual behavior, 11.7% admitted that their actual behavior is quite different from the Internet behavior, and 24.9% admitted that their real-world behavior is completely different from Internet behavior. In the virtual environment of the Internet, it is easy for people to behave differently from the real world. That is, most college students have different knowledge and actions in the network environment.

Therefore, at present, the problems of college students' online moral behavior are (1) lack of online moral knowledge, (2) vague network values, and (3) inconsistent knowledge and action in cyberspace. The reasons for these problems can be summarized as three points: (1) the factors of college students themselves are the root causes; college students have a strong ability to receive information, but their awareness of identifying information is poor; (2) it is influenced by Internet construction status; the formulation of the code of conduct on the Internet cannot keep up with the development of the Internet; and (3) the construction of the network morality education team needs to be strengthened, and the content of network morality education is lacking.

## 4. Conclusion

IPE has long dominated Chinese higher education. Under the background of the new era, it is necessary to do a good job in the online moral education of college students. In the process of online moral education for college students, not only the efforts of colleges and universities but also the joint efforts of the government and society are needed to gather forces from multiple parties to study the road of integration to further accelerate the process of college students' online moral education. Based on the development history of IPE, the online moral behavior of college students is analyzed and studied. The innovation lies in the introduction of CNN, which is convenient for time-series data processing in the data analysis process to improve the accuracy of the output results and increase the objective credibility of the research. The results show that 80.1% of the students do not care about the development of online moral education courses. Among them, 5.1% said they hated the course. The proportion of students who understand or have received cybersecurity education is less than 20%. A considerable part of the subjects did not think that browsing pornographic websites, cyber-attacks, and human flesh searches were unreasonable. Almost all the subjects believed that their real-life behaviors differed from Internet behaviors. This study investigates college students' perceptions of online ethics education. The concept of online moral behavior and students' behavior is used to analyze and judge the current online moral behavior of college students and provide a certain reference for the subsequent research and analysis of online moral behavior education in colleges and universities. The inadequacy lies in the fact that fewer objects are involved in the questionnaire survey, and the data selection range is small. The conclusions of the experimental analysis are only applicable to college students in the surveyed area, and it remains to be further verified whether it is also applicable to other areas. Additionally, it is necessary to conduct in-depth research on whether there are differences in online moral behavior among students of different genders, ages, and majors.

## Figures and Tables

**Figure 1:** Operational structure of CNN.

**Figure 2:** Basic structure diagram of RNN.

**Figure 3:** Grade distribution of respondents.

**Figure 4:** Subject distribution of respondents.

**Figure 5:** Flow of research work.

**Figure 6:** Results of a survey on students' perceptions of online education.

**Figure 7:** Survey results for being educated on ethical behavior online.

**Figure 8:** Survey results of online moral values.

**Figure 9:** Survey results on ethical online behavior.

**Table 1:** Classification of DL algorithms.

DL algorithms	Introduction
Convolution neural network (CNN)	Neural network system based on convolution operation
Deep belief network (DBN)	Pretraining in the form of a multilayer self-encoding neural network and then combined with discriminant information to further optimize the deep belief network of neural network weights
Recurrent neural network (RNN)	Self-encoding neural networks based on multilayer neurons, including autoencoder and sparse coding, have received extensive attention in recent years

## Data Availability

The data used to support the findings of this study are available from the corresponding author upon request.
